The article "Spice Up Your Life: Adipose Tissue and Inflammation" was published in 2014. Journal: J Lipids.

# Spice Up Your Life: Adipose Tissue and Inflammation

**DOI:** 10.1155/2014/182575

**Published:** 2014-02-20

**Authors:** Anil K. Agarwal

**Affiliations:** Division of Nutrition and Metabolic Diseases, Center for Human Nutrition, Department of Internal Medicine, University of Texas Southwestern Medical Center, 5323 Harry Hines Boulevard, Dallas, TX 75390, USA

## Abstract

Cells of the immune system are now recognized in the adipose tissue which, in obesity, produces proinflammatory chemokines and cytokines. Several herbs and spices have been in use since ancient times which possess anti-inflammatory properties. In this perspective, I discuss and propose the usage of these culinary delights for the benefit of human health.

## 1. Introduction

Up until recently, studies relating to adipose tissue were mostly neglected partly because adipose tissue (AT) was not considered to be a critical tissue, except for the fact that AT stores energy (as triglycerides) and releases it upon demand and partly because lipids are very hydrophobic in nature and are not easily soluble in aqueous solutions, further hampering biochemical analysis. Even now, most investigators still use the solvent system developed in 1950 by Bligh and Dyer, is a rapid chloroform and methanol lipid extraction method, although this extraction method is only efficient in extracting some, but not all, types of lipids.

Adipose tissue regained scientific attention in early 1980 with the rise of obesity worldwide [1]. The occurrence of obesity has continued to increase at such a pace that recently it has been classified as a disease by the American Medical Association [2]. While obesity in humans had been described in ancient literature, those who lacked AT went unnoticed. The first documented evidence of a lack of AT in humans was described by Berardinelli and Seip in 1954, who observed patients with complete loss of AT from birth [3, 4]. Since then, several investigators have identified a spectrum of the AT loss, ranging from partial to total, and has been referred to as partial lipodystrophy (PL) and congenital generalized lipodystrophy (CGL), respectively [5–7]. However, when present, AT has the potential to expand up to 50–70% of body weight causing obesity. Ironically, the clinical burden or symptoms in both of these conditions—obesity and lipodystrophy—are quite similar. Patients of both conditions suffer from hypertriglyceridemia, insulin resistance, hepatic steatosis, and development of type 2 diabetes, and in women both conditions may contribute towards polycystic ovarian syndrome (PCOS). These constellations of clinical features are also referred to as Metabolic Syndrome. Because of this, it has become apparent that AT is important for normal physiological function in the human body but may not be critical for human development and survival.

In any human population, there is a continuum of body mass, ranging from extremely lean to lean to obese and extremely obese, resulting in a bell-shaped curve (Figure 1(a)). Thus, on the extreme ends of the graph lies a set of individuals whose AT is most likely regulated by genetic alterations. Such is the case in individuals with CGL, who have germ line transmission of mutations in genes such as 1-acylglycerol 3-phosphate-O-acyltransferase 2 (*AGPAT2*) [8], Berardinelli Seip congenital lipodystrophy 2 (*BSCL2*) [9], and Caveolin 1 (*CAV1*) [10]. At the other end of the spectrum lies the case of extreme obesity, mostly since birth, and here again germ line transmission in genetic alterations was noted in leptin (*LEP*), leptin receptor (*LEPR*), proopiomelanocortin (*POMC*), prohormone convertase 1 (*PCSK1*), melanocortin 4 receptor (*MC4R*), single-minded homolog 1 (*SIM1*), brain-derived neurotrophic factor (*BDNF*), and its receptor TrkB coded by neurotrophic tyrosine kinase receptor type 2 gene (*NTRK2*) reviewed in [11]. Some cases of obesity, like those due to mutations in the leptin gene, can be treated with leptin replacement [12]. Others, such as those due to *MC4R,* which acts at the central nervous system, have been difficult. Likewise, subjects with lipodystrophy who lack leptin have also been successfully treated with leptin replacement therapy [13]. However, these extreme cases of AT loss or excess are extremely rare. It is the vast majority of the human population who fall under the bell-shaped “obesity curve” that require treatment because obesity is associated with a number of chronic diseases like fatty liver (hepatic steatosis), hyperlipidemia, hypercholesterolemia, cardiovascular diseases, and type II diabetes. Obesity in this group appears to be of polygenic nature. Numerous genomewide association studies (GWAS) have identified several single nucleotide polymorphisms (SNPs) enriched in several genes, both in the coding and noncoding regions associated with obesity. These SNPs are too numerous to mention here and are reviewed in [14]. One among them is obesity-associated gene (*FTO*). FTO demethylates N^6^-methyladenosine, a potential regulatory RNA modification, has recently been shown to regulate ghrelin, a hunger hormone, which predisposes to increased food intake and increases obesity [15]. It has also been observed that survivors of childhood brain cancers have a higher risk of developing obesity. A prospective study, *CanDECIDE* study (Canadian Study of Determinants of Endometabolic Health in CHI1DrEn) has been proposed to determine the mechanism(s) associated with inflammation, childhood brain cancer, and the development of obesity [16]. From these observations, it is clear that either losing AT or acquiring excess AT is both unacceptable strategies. Thus, maintaining an adequate amount of healthy AT seems to be a reasonable and acceptable possibility. There are several options for this group of individuals, although adopting a healthy diet and exercise program, when followed, is the most viable option.

## 2. Adipose Tissue

In recent years, interest in AT has seen a renaissance. There have been studies which show that AT (specifically adipocytes), in addition to storing and releasing fatty acid, also secretes several proteins which act as hormones [17]. In addition, AT also secretes lipids which help to maintain systemic metabolic homeostasis [18]. However, adipocytes are not the only cell type which constitutes AT. In addition, AT also contains stromal cells, vascular cells, and cells of the immune system like macrophages [19], specifically of the M2 type, which are anti-inflammatory in lean AT. Several proteins are secreted from adipocytes, often known as adipokines, but the two most widely studied adipokines are leptin [20] and adiponectin [21]. During obesity, AT expands, attracting other cell types; the most important in recent years are the cells of the immune system.

## 3. Anatomical Location of Adipose Tissue

In humans and rodents, AT is found in almost all anatomical regions of the body. It is interesting to note that, unlike other organs such as the liver, heart, or lung, the AT lacks a well-defined organ boundary and thus is mainly identified by anatomical location [29]. AT found under the skin or dermis is mainly referred to as subcutaneous (sc) adipose tissue. AT can further be identified as sc abdominal or sc AT of the extremities. The AT found in the visceral cavity may be subdivided as omental, mesenteric, or perirenal [29]. Adipose tissue located behind the eyes (retroorbital), knees (periarticular), around the hip joints, or beneath the skull has not received any specific nomenclature as yet. While the white AT is distributed throughout the body, the other type of AT—the brown adipose tissue (BAT)—is more restricted in its anatomical location and is mainly found in the interscapular and cervical (neck) region. In the past, BAT was mainly recognized neonatally and in infants and was thought to recede during adulthood. In recent years, new imaging techniques have identified that BAT still exists in the adult human population. While the physiological function of subcutaneous and visceral AT is widely studied, AT found at other locations has received little attention. However, identification of adult BAT has rejuvenated studies related to the physiological function of BAT.

## 4. Types of Adipose Tissue

In the past, two main types of ATs were described—WAT and BAT. Regardless of WAT localization, the WAT has been implicated in maintaining lipid homeostasis. The adipocytes in WAT are insulin sensitive and, thus, in the presence of excess fatty acid, synthesize TAG. These molecules are stored as large lipid droplets in the adipocytes. WAT then releases free fatty acids as required. In contrast, BAT is mainly associated with thermogenesis. The adipocytes of BAT are rich in uncoupling protein 1 (Ucp1) which uncouples the last step in mitochondrial oxidation of fatty acid to release energy instead of generating ATP for storage. In recent years, a new type of adipocyte has been identified, referred to as a “brite” adipocyte (brown-in-white) [30]. Using lineage-tracing reporter mice, Ucp1 promoter-driven GFP for transient tracing of UCP1 expression and UCP1-CreER, ROSA-tdRFP mice to permanently label brown and brite adipocytes following tamoxifen administration, Rosenwald et al. revealed that the origin of brite adipocytes lies in the white adipocytes [31]. Furthermore, this study also revealed that this conversion of white to brite is a reversible process as well.

## 5. Immune Cells of Adipose Tissues

The relationship between the immune system and AT was recognized several decades ago when it was shown that neutralizing tumor necrosis factor alpha (TNF*α*) improved insulin resistance in rodents [19]. This observation catalyzed our thoughts towards systemic inflammation and its role in insulin resistance and obesity. Immune cells of both innate and adaptive immune systems are found in AT obtained from both lean and obese subjects [32]. These include, but are not limited to, macrophages (M1 and M2), mast cells, neutrophils, eosinophils, type 2 innate lymphoid cells (ILCs), CD4+ and CD8+ T cells, B cells, regulatory T (Treg) cells, and natural killer T cells (NKT cells) [32]. In the lean AT, the macrophages are of the M2-type which are anti-inflammatory [33]. It is upon expansion of AT that there is a significant increase in the number of proinflammatory macrophages denoted M1-type [34]. Based on cell surface markers, a new population of adipose tissue macrophage has been identified as type 3 [35], but its role in adipose tissue in relation to M1 and M2 remains to be established. The conversion of the anti-inflammatory M2-type to the proinflammatory M1-type is regulated by lipopolysaccharide and interferon *γ* (IFN-*γ*) which produce proinflammatory mediators like TNF-*α*, IL-6, IL-1*β*, nitric oxide (NO), and IL-12 (Figure 1(b)). While such events in obesity are recognized by several investigators, it is still unclear how the expanding adipose tissue in obese individuals recruits these cells of the immune system.

While the ligands for the cellular triggering of the proinflammatory immune cells can be varied, most of the signal transduction is related via the activation of nuclear factor-kappa B (NF-*κ*B). NF-*κ*B has many members which include REL family members RELA (p65), c-REL and RELB, NF-*κ*B1 (p50; p105), and NF-*κ*B2 (p52; p100). These proteins contain dimerization and DNA-binding domains and can form homo- or heterodimers. NF-*κ*B resides in the cytoplasm and exists as a p50-p65 or p52-p65 dimer associated with the regulatory proteins inhibitor of nuclear factor *κ*B (I*κ*B) kinases (IKKs) [36]. This association with IKKs precludes the complex from entering the nucleus. Upon proinflammatory signals, IKK phosphorylates IkB which then dissociates itself from the p50-p65 or p52-p65 complex and is degraded via ubiquitination, while NF-*κ*B moves into the nucleus to activate the proinflammatory gene program, reviewed in [37]. There are at least four IKKs: IKK-*α*, IKK-*β*, IKK-*ε*, and TANK-binding kinase 1 (TBK1). Recently, it was demonstrated that in vivo inhibition of TBK1 and IKK-*ε* using the small-molecule selective inhibitor amlexanox in mice fed high-fat diet improved insulin sensitivity and decreased hepatic steatosis with accompanying increased energy expenditure and weight loss [38]. This provides a rationale for the effective use of anti-inflammatory molecules for reducing inflammatory-associated obesity and its associated complications.

## 6. Combating Inflammation in Obesity and Metabolic Syndrome

Ever since the identification of the role of low grade inflammation in obesity and its associated complications, efforts have been underway to reduce the burden of inflammation in AT. Thus, reducing the proinflammatory response in AT should be beneficial for human health.

Several phytochemicals have been in use since prehistoric times, although the anti-inflammatory properties of these culinary herbs and spices were only recognized recently. These phytochemicals belong to several chemical groups but most belong to polyphenols, flavonoids and their analogs. When consumed in small quantities, certain plants, including plant roots themselves and their extracts, have been reported to have beneficial effects in reducing systemic inflammation and type 2 diabetes and increasing insulin sensitivity. A recent report shows that high-fat fed mice given dietary capsaicin, a component of chili pepper, showed improved glucose tolerance, reduced liver fat, and improved insulin sensitivity [39]. In another study, the topical application of capsaicin in mice saw a reduction in visceral adipose tissue resulting in decreased inflammation and increased insulin sensitivity [40]. Capsaicinoids, a group of chemicals found in chili pepper, have also been shown to have a beneficial effect on weight loss in humans [41]. This effect has been shown to be due to increased energy expenditure, increased lipid oxidation, and decrease in appetite [41]. A meta-analysis of the use of capsaicinoids further confirms their role in weight loss [42]. However, further investigations are needed to evaluate their role in long-term usage. Although it is unclear what role capsaicin plays in cancer, studies with capsaicin extract, which is a mixture of several molecules, including norhydrocapsaicin, dihydrocapsaicin, homocapsaicin, homodihydrocapsaicin, and nonivamide, have resulted in showing both the carcinogenic and anticarcinogenic activities of capsaicin (reviewed in [43]). Why capsaicin has demonstrated both activities might be due to the fact that various capsaicin extracts used in the studies do not carry the same chemical entities or might vary in the concentration of various chemical components or because of their different metabolism rates in humans and animals [43, 44].

The role of natural products in cachexia has not been fully elucidated. This is partly because there is a lack of consensus as to how to define cachexia. A recent attempt defines cancer cachexia as “…ongoing loss of skeletal muscle mass with or without loss of fat mass that cannot be reversed by conventional nutritional support and leads to progressive functional impairment” [45, 46]. In fact, both cachexia and obesity, which represent two different nutritional states, have some similarities in expression of inflammatory molecules. IL-6 and TNF are expressed in both conditions. However, in obesity, additional proinflammatory molecules IL-1*β* and interferon *γ* are also expressed. I hypothesize that the use of some of the anti-inflammatory products derived from the plant source might result in beneficial effects for these patients [47]. I have discussed genetic causes of lipodystrophy and, by itself, loss of adipose tissue does not attract cells of the immune system. However, the advent of highly active antiretroviral therapy (HAART) for the treatment of patients affected with human immunodeficiency virus (HIV) did result in partial lipodystrophy. Although lack of adipokines such as leptin or adiponectin [48] has been reported, information regarding cells of the immune system is scarce and treatment with plant derived products is yet to take hold.

I have listed in Table 1 several of these plants and roots which have been used in many cultures to enhance the food flavors. In the process, these cultures have also benefitted from their anti-inflammatory properties, which have been extensively reviewed in [22, 26, 49, 50]. This is not to say that consuming all of these spices will make the obesity-associated inflammation go away, but they will help alleviate some of its effects. A sustained but balanced diet and exercise is still required to combat obesity and associated inflammation. There are no systematic controlled clinical trials using these spices and herbs to further provide the rationale for using these spices for this purpose. This is partly because these phytochemicals are often not extracted, purified, and identified as a single chemical entity and partly because these phytochemicals vary according to the geographic location which further makes the outcome of these studies scientifically unreliable. However, these herbs and spices have been used from prehistoric times with beneficial effects. Another aspect to consider is that while one single spice might bring a small biological effect, when used in combination with a mixture of spices, they might show additive effects. Therefore, while controlled clinical trials might improve our confidence in the usage of these spices, nevertheless, their usage in crude form in our daily lives will still bring benefits.

## 7. Brown Adipose Tissue and Inflammation

I have discussed above the physiological function of BAT in human physiology which is to provide thermogenic activity by the uncoupling of energy which has been proposed as a mechanism to alleviate obesity. In humans, BAT was thought to be present in infants but not in adults. All this changed with the improvements in detection technology. BAT actively uptakes glucose from the blood. Thus, detecting glucose using a noninvasive technique coupled with the presence of UCP1, a molecular signature for BAT should yield the presence of BAT in adult humans. When ^18^F-fluorodeoxyglucose (^18^F-FDG) positron-emission tomographic and computed tomographic (PET-CT) scans were performed, significant depots of BAT was revealed from the anterior neck to the thorax region in human adults [51]. Therefore, activating BAT in human adults seems to be approachable now. The role of alternatively activated macrophages in the control of BAT thermogenesis was recently demonstrated in rodents by Nguyen et al. [52], suggesting for the first time the relationship between cells of the immune system and BAT. While searching for alternative ways to activate BAT, Zhu et al. [53] discovered the expression of transient receptor potential melastin 8 (TRPM8), a cold sensing ion channel, which responded to menthol in inducing BAT thermogenesis. Transient receptor potential vanilloid-4 (TRPV4) has also been found to be expressed in the BAT and is believed to be the inhibitor of the molecular function of beige adipose tissue. Thus, inhibition of TRPV4 leads to an increase in the thermogenic gene expression in WAT [54]. In addition to BAT, TRPV4 is also present in sympathetic nervous system (SNS) which could further regulate BAT. The physiological ligand for TRPV4 is still unknown but has provided new avenues for regulation BAT.

It is also interesting to note that several of the ion channels expressed in our palate are activated by compounds present in our food. The taste cells on the tongue, throat, and mouth synapse with adherent fibers that travel to the brain via the trigeminal nerve. In addition to TRPV4 and TRPM8 as found in BAT, these nerves express other ion channels such as transient receptor potential V1 (TRPV1, TRPA1, and TRPV3). These TRP-types of channels are activated by alkamides, isothiocyanates, and terpene dialdehydes found in the diet we consume. Although most spices, such as capsaicin, piperazine, chili, and rutaecarpine—found in a Chinese herb (Wu-Chu-Tu) [55], have been found to activate TRP1 in the palate, it is possible that they might activate other ion channels. Therefore, these spices might have benefits in activating BAT in addition to flavoring our food. Indeed, a recent study demonstrated the beneficial effect of capsinoids when ingested by humans for over a 6-week period, increasing energy expenditure and reducing body fat [56].

## 8. Characterization of Natural Products

Despite the fact that we recognize the beneficial effects of plant products, identifying the active ingredient has been challenging. First, geographic location and the prevailing climate conditions can alter the chemical composition of the active substance. In fact, such variation can be noted from season to season within the same geographic location. Second, the very extraction method employed, while this might be optimized, could also alter the chemical composition of the active substance. Third, the fact that each plant extract consists of several individual chemically distinct compounds further complicates the isolation of a single active compound.

## 9. Perspective

Overall, the purpose of this perspective is to advance the idea of the beneficial effect of spices used in all cultures—some more than others—including their effects in alleviating inflammation, a partner in obesity causing associated metabolic complications. A recent study demonstrated the beneficial effect of curcumin, the active substance of turmeric, as an effective treatment for inflammatory bowel disorder [57]. Salicylate, or its acetylated form, aspirin, is the oldest and most widely prescribed drug first identified in plants [58]. Its effect in lowering blood glucose was first reported by Yuan et al. [59, 60]. Salsalate's beneficial effect was recently reported in placebo-controlled, randomized clinical trial [61, 62]. Although controlled clinical trials for many of the phytochemicals are not feasible for the reasons mentioned above, more efforts are needed to isolate and identify the chemical entity and biological activity of phytochemicals as has been demonstrated for curcumin and salsalate.

## Figures and Tables

**Figure 1:** Schematic of body fat in a human population and the presence of macrophages in lean and obese adipose tissue. (a) The bell-shaped curve represents the distribution of body fat in a human population. The healthy weight (within the 1 standard deviation of the healthy weight) is shown between the black dashed lines. In recent decades, this curve has shifted to the right, shown by the diagonal shaded red lines. The increase in this body weight is also associated with various single nucleotide polymorphisms found in the general population. On the extreme ends, monogenic forms of congenital generalized lipodystrophy (CGL) and obesity are shown in the circles. Various genes associated with these monogenic forms are mentioned in the text. (b) Anti-inflammatory M2 macrophages in the lean adipose tissue are converted to proinflammatory M1 macrophages in the obese adipose tissue which depends on chronic nutrition, chemokine, and cytokine signaling.

**Table 1:** Shown are some of the more commonly used herbs and spices, possible active ingredients, and anti-inflammatory mechanisms. This is not an exhaustive list of herbs and spices but is used to illustrate the beneficial effects of these herbs and spices. For many, the entire range of active ingredients is unknown and most are used in powder form or as an aqueous extract. A few are used as an oil extract.

Common name	Botanical name	Anti-inflammatory properties	Possible mechanism	Active ingredient	Reference
Allspice	*Pimenta officinalis/Pimenta dioica *	Yes	N.D.		[22]
Anise	*Pimpinella anisum *	Yes	↓NF-*κβ*	Anethol	[23]
Bay leaf	*Laurus nobilis *	Yes		Quercetin	[22]
Black pepper	*Piper nigrum *	Yes	↓adipogenesis	Piperine	[24, 25]
Caraway	*Carum carvi *	Yes	N.D.	Aqueous extract	[22]
Chili pepper	*Capsicum annuum L. *	Yes	↓NF-*κβ* by blocking I*κ*B*α* degredation	Capsaicin	[26]
Cinnamon	*Cinnamomum cassia *	Yes	N.D.	Benzyl cinnamide/cinnamic acid	[22]
Clove	*Syzygium aromaticum *	Yes	↓Cox-2	Carvacrol/eugenol	[25]
Cocoa	*Theobroma cacao (seed) *	Yes	↓NF-*κβ* ↓adipogenesis	Catechin, mixture of several flavanols	[26]
Coriander	*Coriandrum sativum *	Yes	Antioxidant	Galic acid/seed or plant extract	[26]
Cumin	*Cuminum cyminum *	Yes	N.D.	Cuminaldehyde, cumin oil, oleorestin	[26]
Fenugreek	*Trigonella foenum-graecum *	Yes	N.D.	Used as extract	[26]
Ginger	*Zingiber officinale (underground stem) *	Yes	↓NF-*κβ* ↓Cox-2	6-Gingerol, 10-gingerol, shogaol	[27]
Marjoram	*Origanum majorana *	Yes	N.D.	Rosmarinic	[28]
Oregano	*Origanum vulgare *	Yes	↓Cox-2	Biochanin A/diosmetin	[28]
Rosemary	*Rosmarinus officinalis *	Yes	N.D.	Rosmarinic/luteolin	[28]
Sage	*Salvia officinalis *	Yes	↓Cox-2	Rosmarinic/apigenin	[28]
Soy/soy beans	*Glycine max *	Yes	↓NF-*κβ*	Genistein	[26]
Thyme	*Thymus vulgaris *	Yes	↓Cox-2	Rosmarinic/luteolin	[28]
Turmeric	*Curcuma longa *	Yes	↓NF-*κβ* ↑apoptosis	Curcumin (aka curcuminoids)	[27]

N.D.: not determined; aka: also known as; NF-*κβ*: nuclear factor kappa B; Cox-2: cyclooxygenase isoform 2; ↓: decrease in activity; ↑: increase in activity.

## References

[1] Finucane MM, Stevens GA, Cowan MJ (2011). National, regional, and global trends in body-mass index since 1980: Systematic analysis of health examination surveys and epidemiological studies with 960 country-years and 9*·*1 million participants. *The Lancet*.

[2] http://www.ama-assn.org/assets/meeting/2013a/a13-addendum.pdf.

[3] Berardinelli W (1954). An undiagnosed endocrinometabolic syndrome: report of 2 cases. *The Journal of Clinical Endocrinology and Metabolism*.

[4] Seip M (1959). Lipodystrophy and gigantism with associated endocrine manifestations. A new diencephalic syndrome?. *Acta Paediatrica*.

[5] Agarwal AK, Garg A (2006). Genetic disorders of adipose tissue development, differentiation, and death. *Annual Review of Genomics and Human Genetics*.

[6] Garg A (2011). Lipodystrophies: genetic and acquired body fat disorders. *Journal of Clinical Endocrinology and Metabolism*.

[7] Vantyghem MC, Balavoine AS, Douillard C (2012). How to diagnose a lipodystrophy syndrome. *Annales D Endocrinologie*.

[8] Agarwal AK, Arioglu E, De Almeida S (2002). AGPAT2 is mutated in congenital generalized lipodystrophy linked to chromosome 9q34. *Nature Genetics*.

[9] Magré J, Delépine M, Khallouf E (2001). Identification of the gene altered in Berardinelli-Seip congenital lipodystrophy on chromosome 11q13. *Nature Genetics*.

[10] Kim CA, Delépine M, Boutet E (2008). Association of a homozygous nonsense caveolin-1 mutation with berardinelli-seip congenital lipodystrophy. *Journal of Clinical Endocrinology and Metabolism*.

[11] Ramachandrappa S, Farooqi IS (2011). Genetic approaches to understanding human obesity. *Journal of Clinical Investigation*.

[12] Farooqi IS, Jebb SA, Langmack G (1999). Effects of recombinant leptin therapy in a child with congenital leptin deficiency. *The New England Journal of Medicine*.

[13] Oral EA, Simha V, Ruiz E (2002). Leptin-replacement therapy for lipodystrophy. *The New England Journal of Medicine*.

[14] Choquet H, Meyre D (2011). Molecular basis of obesity: current status and future prospects. *Current Genomics*.

[15] Efthimia K, O'Daly OG, Choudhury AI (2013). A link between FTO, ghrelin, and impaired brain food-cue responsity. *The Jouranl of Clinical Investigation*.

[16] Samaan MC, Thabane L, Burrow S, Dillenburg RF, Scheinemann K (2013). Canadian Study of Determinants of Endometabolic Health in ChIlDrEn (CanDECIDE study): a cohort study protocol examining the mechanisms of obesity in survivors of childhood brain tumours. *British Medical Journal*.

[17] Alvarez-Llamas G, Szalowska E, de Vries MP (2007). Characterization of the human visceral adipose tissue secretome. *Molecular and Cellular Proteomics*.

[18] Cao H, Gerhold K, Mayers JR, Wiest MM, Watkins SM, Hotamisligil GS (2008). Identification of a lipokine, a lipid hormone linking adipose tissue to systemic metabolism. *Cell*.

[19] Hotamisligil GS, Shargill NS, Spiegelman BM (1993). Adipose expression of tumor necrosis factor-*α*: direct role in obesity-linked insulin resistance. *Science*.

[20] Zhang Y, Proenca R, Maffei M, Barone M, Leopold L, Friedman JM (1995). Correction: positional cloning of the mouse obese gene and its human homologue. *Nature*.

[21] Li S, Shin HJ, Ding EL, Van Dam RM (2009). Adiponectin levels and risk of type 2 diabetes: a systematic review and meta-analysis. *Journal of the American Medical Association*.

[22] Jungbauer A, Medjakovic S (2012). Anti-inflammatory properties of culinary herbs and spices that ameliorate the effects of metabolic syndrome. *Maturitas*.

[23] Rajput S, Mandal M (2012). Antitumor promoting potential of selected phytochemicals derived from spices: a review. *European Journal of Cancer Prevention*.

[24] Park U-H, Jeong H-S, Jo E-Y (2012). Piperine, a component of black pepper, inhibits adipogenesis by antagonizing PPAR*γ* activity in 3T3-L1 cells. *Journal of Agricultural and Food Chemistry*.

[25] Mueller M, Beck V, Jungbauer A (2011). PPAR*α* activation by culinary herbs and spices. *Planta Medica*.

[26] Siriwardhana N, Kalupahana NS, Cekanova M, LeMieux M, Greer B, Moustaid-Moussa N (2013). Modulation of adipose tissue inflammation by bioactive food compounds. *The Journal of Nutritional Biochemistry*.

[27] Ramadan G, Al-Kahtani MA, El-Sayed WM (2011). Anti-inflammatory and anti-oxidant properties of curcuma longa (turmeric) versus Zingiber officinale (ginger) rhizomes in rat adjuvant-induced arthritis. *Inflammation*.

[28] Park JB (2011). Identification and quantification of a major anti-oxidant and anti-inflammatory phenolic compound found in basil, lemon thyme, mint, oregano, rosemary, sage, and thyme. *International Journal of Food Sciences and Nutrition*.

[29] Simha V, Agarwal AK (2007). *Inherited and Acquired Lipodystrophies; Disorders of Adipose Tissue Development, Differentiation, and Death*.

[30] Wu J, Bostrom P, Sparks LM (2012). Beige adipocytes are a distinct type of thermogenic fat cell in mouse and human. *Cell*.

[31] Rosenwald M, Perdikari A, Rulicke T, Wolfrum C (2013). Bi-directional interconversion of brite and white adipocytes. *Nature Cell Biology*.

[32] Mathis D (2013). Immunological goings-on in visceral adipose tissue. *Cell Metabolism*.

[33] Chawla A, Nguyen KD, Goh YPS (2011). Macrophage-mediated inflammation in metabolic disease. *Nature Reviews Immunology*.

[34] Lumeng CN, Bodzin JL, Saltiel AR (2007). Obesity induces a phenotypic switch in adipose tissue macrophage polarization. *Journal of Clinical Investigation*.

[35] Zeyda M, Gollinger K, Kriehuber E, Kiefer FW, Neuhofer A, Stulnig TM (2010). Newly identified adipose tissue macrophage populations in obesity with distinct chemokine and chemokine receptor expression. *International Journal of Obesity*.

[36] Li Q, Verma IM (2002). NF-*κ*B regulation in the immune system. *Nature Reviews Immunology*.

[37] Chau T-L, Gioia R, Gatot J-S (2008). Are the IKKs and IKK-related kinases TBK1 and IKK-*ε* similarly activated?. *Trends in Biochemical Sciences*.

[38] Reilly SM, Chiang SH, Decker SJ (2013). An inhibitor of the protein kinases TBK1 and IKK-varepsilon improves obesity-related metabolic dysfunctions in mice. *Nature Medicine*.

[39] Kang J-H, Tsuyoshi G, Han I-S, Kawada T, Kim YM, Yu R (2010). Dietary capsaicin reduces obesity-induced insulin resistance and hepatic steatosis in obese mice fed a high-fat diet. *Obesity*.

[40] Lee GR, Shin MK, Yoon DJ (2013). Topical application of capsaicin reduces visceral adipose fat by affecting adipokine levels in high-fat diet-induced obese mice. *Obesity*.

[41] Whiting S, Derbyshire E, Tiwari BK (2012). Capsaicinoids and capsinoids. A potential role for weight management? A systematic review of the evidence. *Appetite*.

[42] Whiting S, Derbyshire EJ, Tiwari B (2014). Could capsaicinoids help to support weight management? A systematic review and meta-analysis of energy intake data. *Appetite*.

[43] Bley K, Boorman G, Mohammad B, McKenzie D, Babbar S (2012). A comprehensive review of the carcinogenic and anticarcinogenic potential of capsaicin. *Toxicologic Pathology*.

[44] Richter E, Engl J, Friesenegger S, Tricker AR (2009). Biotransformation of 4-(methylnitrosamino)-1-(3-pyridyl)-1-butanone in lung tissue from mouse, rat, hamster, and man. *Chemical Research in Toxicology*.

[45] Argilés JM, Anker SD, Evans WJ (2010). Consensus on cachexia definitions. *Journal of the American Medical Directors Association*.

[46] Fearon KCH (2011). Cancer cachexia and fat-muscle physiology. *The New England Journal of Medicine*.

[47] Tsoli M, Robertson G (2013). Cancer cachexia: malignant inflammation, tumorkines, and metabolic mayhem. *Trends in Endocrinology and Metabolism*.

[48] Paruthi J, Gill N, Mantzoros CS (2013). Adipokines in the HIV/HAART-associated lipodystrophy syndrome. *Metabolism*.

[49] Gosslau A, Li S, Ho C-T, Chen KY, Rawson NE (2011). The importance of natural product characterization in studies of their anti-inflammatory activity. *Molecular Nutrition and Food Research*.

[50] Leiherer A, Mundlein A, Drexel H (2013). Phytochemicals and their impact on adipose tissue inflammation and diabetes. *Vascular Pharmacology*.

[51] Cypess AM, Lehman S, Williams G (2009). Identification and importance of brown adipose tissue in adult humans. *The New England Journal of Medicine*.

[52] Nguyen KD, Qiu Y, Cui X (2011). Alternatively activated macrophages produce catecholamines to sustain adaptive thermogenesis. *Nature*.

[53] Zhu Z, Ma S, Yu H (2012). Activation of the cold-sensing TRPM8 channel triggers UCP1-dependent thermogenesis and prevents obesity. *Journal of Molecular Cell Biology*.

[54] Ye L, Kleiner S, Wu J (2012). TRPV4 is a regulator of adipose oxidative metabolism, inflammation, and energy homeostasis. *Cell*.

[55] Nilius B, Appendino G (2011). Tasty and healthy TR(i)Ps. the human quest for culinary pungency. *The EMBO Reports*.

[56] Yoneshiro T, Aita S, Matsushita M (2013). Recruited brown adipose tissue as an antiobesity agent in humans. *The Journal of Clinical Investigation*.

[57] Baliga MS, Joseph N, Venkataranganna MV, Saxena A, Ponemone V, Fayad R (2012). Curcumin, an active component of turmeric in the prevention and treatment of ulcerative colitis: preclinical and clinical observations. *Food Function*.

[58] Jack DB (1997). One hundred years of aspirin. *The Lancet*.

[59] Yuan M, Konstantopoulos N, Lee J (2001). Reversal of obesity- and diet-induced insulin resistance with salicylates or targeted disruption of Ikk*β*. *Science*.

[60] Kim JK, Kim Y-J, Fillmore JJ (2001). Prevention of fat-induced insulin resistance by salicylate. *Journal of Clinical Investigation*.

[61] Goldfine AB, Fonseca V, Jablonski KA, Pyle L, Staten MA, Shoelson SE (2010). The effects of salsalate on glycemic control in patients with type 2 diabetes: a randomized trial. *Annals of Internal Medicine*.

[62] Goldfine AB, Fonseca V, Jablonski KA, Pyle L, Staten MA, Shoelson SE (2010). The effects of salsalate on glycemic control in patients with type 2 diabetes: a randomized trial. *Annals of Internal Medicine*.

